The article "Increasing power generation to a single-chamber compost soil urea fuel cell for carbon-neutral bioelectricity generation: A novel approach" was published in 2023. Journal: Front Microbiol.

# Increasing power generation to a single-chamber compost soil urea fuel cell for carbon-neutral bioelectricity generation: A novel approach

**DOI:** 10.3389/fmicb.2023.1086962

**Published:** 2023-02-17

**Authors:** Verjesh Kumar Magotra, Dong-Jin Lee, D. Y. Kim, S. J. Lee, T. W. Kang, Arjun Magotra, Akbar I. Inamdar, Nabeen K. Shrestha, Supriya A. Patil, Siriluck Thammanu, Hee Chang Jeon

**Affiliations:** ^1^Quantum-Functional Semiconductor Research Center, Dongguk University, Seoul, Republic of Korea; ^2^Department of Computer Science and Engineering, Dongguk University, Seoul, Republic of Korea; ^3^Division of Physics and Semiconductor Science, Dongguk University, Seoul, Republic of Korea; ^4^Department of Nano Technology and Advanced Materials Engineering, Sejong University, Seoul, Republic of Korea; ^5^Royal Forest Department, Bangkok, Thailand

**Keywords:** carbon-neutral, urea fuel cell, carbon-rich compost soil, wastewater, energy

## Abstract

Microbial fuel cells (CS-UFC) utilize waste resources containing biodegradable materials that play an essential role in green energy. MFC technology generates “carbon-neutral” bioelectricity and involves a multidisciplinary approach to microbiology. MFCs will play an important role in the harvesting of “green electricity.” In this study, a single-chamber urea fuel cell is fabricated that uses these different wastewaters as fuel to generate power. Soil has been used to generate electrical power in microbial fuel cells and exhibited several potential applications to optimize the device; the urea fuel concentration is varied from 0.1 to 0.5 g/mL in a single-chamber compost soil urea fuel cell (CS-UFC). The proposed CS-UFC has a high power density and is suitable for cleaning chemical waste, such as urea, as it generates power by consuming urea-rich waste as fuel. The CS-UFC generates 12 times higher power than conventional fuel cells and exhibits size-dependent behavior. The power generation increases with a shift from the coin cell toward the bulk size. The power density of the CS-UFC is 55.26 mW/m^2^. This result confirmed that urea fuel significantly affects the power generation of single-chamber CS-UFC. This study aimed to reveal the effect of soil properties on the generated electric power from soil processes using waste, such as urea, urine, and industrial-rich wastewater as fuel. The proposed system is suitable for cleaning chemical waste; moreover, the proposed CS-UFC is a novel, sustainable, cheap, and eco-friendly design system for soil-based bulk-type design for large-scale urea fuel cell applications.

## Introduction

The depletion of fossil fuels and the increase in environmental pollution necessitate energy solutions. Microbial fuel cells (MFCs) utilize waste resources containing biodegradable materials and play an important role in green energy. MFC technology, a “carbon-neutral” bioelectricity generator, involves a multidisciplinary approach to microbiology (Thulasinathan et al., 2022). Environmental awareness has increased the demand for green electricity, which is electricity generated entirely from renewable energy sources (Calikoglu and Koksal, 2022) it has various opportunities and challenges such as electrophysiology, electrochemical, and process engineering (Magotra et al., 2020). MFC technology will play an important role in the harvesting of “green electricity.” Moreover, the rapid increase in power consumption and various environmental issues have compelled the research community to identify new sources of renewable energy (Kumar et al., 2018). MFCs use bacteria or secreted enzymes to break down fuel for power generation. In MFCs, bacteria and enzymes act as biocatalysts for the oxidation and reduction reactions involved in electricity production in compost soil systems (Ziyauddin and Pathrikar, 2013).

Almost all liquid MFCs have associated safety concerns; they quickly degrade due to the volatilization of ammonia, which mainly occurs due to toxicity, shifting, and leakage problems. Therefore, compost soil is preferred over liquid MFCs to minimize degradation risks and enhance microbial activity so that less fuel is consumed as well as to increase the work efficiency and yield more power, as discussed in our previous coin cell studies (Adegoke, 2022). Furthermore, reliable sources are usually cheap and do not cause volatilization issues; moreover, maintaining the pH levels in the soil in a solid state is easy to maintain (Anglada et al., 2010). Among all the available resources of sustainable energy, urea is a suitable fuel for MFCs. Urea application methods are key factors that influence NH_3_ emission either by increase or decrease (Magotra et al., 2022). Advantageously, composting soil microbes during their growth naturally causes nitrification and denitrification in urea (Kapałka et al., 2011). Compost soil is the best electrocatalyst reported in previous studies that are cheap and sustainable (Angar and Eddine, 2015) in this study, we propose the use of stable compost soil and urea-rich waste as fuel for energy generation. Compost soil acts as a mediator, ionic conductor, separator, and source of electro-genic bacteria, which supply additional nutrients to the microbes (Perez et al., 2012; Kumar et al., 2018). The proposed system is a complex system containing water, mineral, and bacteria, which are beneficial for plants too (Burke and Nugent, 1983; Lan, 2010; Teng et al., 2019).

The other advantage of the proposed system is the availability of reliable and leak-proof systems, which are easy to handle. A coin cell system is small, and thus, it is hard for the system to club the powers (Cho and Hoffmann, 2017). Nevertheless, it is easier for bulk single-chamber fuel cells to club the powers at a large scale and makes connections compared to coin cells. The bulk-size design affords many advantages in terms of power and maintenance (Rollinson et al., 2011; Piche-Choquette and Constant, 2019; Vaishali and Das, 2019). Bulk-sized CS-UFC fuel cells can easily refuel with abundant urea waste fuel and can easily prepare stacks in series and parallel for power generation at high rates. Which is not possible in coin cell fuel cells (Bor-Yann et al., 2013).

The coin type size is good for testing by this we can save the waste of material, and research time, easily we can find the way out for testing results and whether the experiment will work or not. Coin cell is mostly used for doing to analyzing the sample performance at a small scale level. We are using a coin cell for initial studies as the best option. The coin cell surface area is very small. As we had discussed that if we increase the size of the surface area from a coin cell (surface area of 3.14 cm^2^) as compared to a single chamber CS-UFC having (a surface area of 15cm^2^), the power density will be enhanced from (coin cell: 3 mW/m^2^ → to the single chamber: 55.27 mW/m^2^). For electrical applications, a coin cell is not a suitable solution for power generation. Either in comparison with stacks in series or parallel circuits. In a single chamber is easy to supply fuel and the lifetime of the fuel cell will also be enhanced due to refueling fuel for a higher power generation system.

Thus, these are novel and promising approaches for generating sustainable green energy at a large scale using any type of urea-rich waste as fuel. MFC technology provides a method for sustainable energy generation (Magotra et al., 2022). It decomposes corrosive substances *via* a “carbon-neutral” process to generate energy from organic waste. This carbon-neutral renewable energy generation technology can realistically replace fossil-fuel-based energy generation technologies that release fixed carbon into the atmosphere. Therefore, it can be used for the sustainable development of humankind (Vraghavulu et al., 2009; Huazhang et al., 2012).

Additionally, CS-UFC applications for recycling and reuse have been technically feasible for reducing CO_2_ in wastewater (per day efficiency of 40–60% relative to formic acid) for bioenergy and material generation. CS-UFCs can consume organic wastewater or waste and convert them into valuable chemicals (e.g., formic acid) to reduce CO_2_ (Wang et al., 2013). CS-UFCs employ catalyst electrodes and bioelectrochemical systems to realize CO_2_ reduction without external energy input, subsequently capturing and converting CO_2_ (Wang et al., 2017).

Urea/urine wastewaters can be treated following an oxidation reaction to release nitrogen gas before their discharge into the environment, or they can be converted to recycled water after further treatment (Boggs et al., 2009).

Herein, a compost soil that uses naturally collected urea-rich wastewater as fuel is supplied to the single chamber CS-UFC. At anode and cathode with the same work, functional graphite electrodes for power generation and environment cleaning were analyzed under different urea concentrations. Further studies were done by selecting using 0.5 g/mL urea fuel concentration. Additionally, this multifunctional CS-UFC was successfully helpful to reduce the toxicity, and pollution, from urea-rich water using soil processes soil based systems, are cheap and trusted for cleaning soil air, and groundwater and safe the environment. This technology itself is clean, safe, and sustainable (Ziyauddin and Pathrikar, 2013; Magotra et al., 2021).

## Methods

### Sample preparation

Compost soil was supplied by Seoul Seung Jin compost soil, Fertilisers Pvt. Ltd., Korea. The compost is carbon-rich soil that was composed of dry leaves and Carbon-rich matter like branches, stems, dried leaves, peels, bits of wood, bark dust or sawdust pellets, shredded brown paper bags, corn stalks, coffee filters, coffee grounds, conifer needles, egg shells, straw, peat moss, wood ash gives compost its light, fluffy body, and decomposed plant products (Singh et al., 2013). Graphite electrodes were used as the anode and cathode. Initial studies were conducted with five different concentrations of urea fuel cells for optimization: 0.1, 0.2, 0.3, 0.4, and 0.5 g/mL, using a single chamber CS-UFC with graphite/graphite (Gr/Gr) as electrodes (Baveye et al., 2020). To compare the power generation, the urea fuel concentration was fixed at 0.5 g/mL in the liquid state and mixed with 50 grams of soil for a bulk fuel cell having a surface area of 15 cm^2^. The Urea-based fuel cell was designed with sustainable properties and optimized conditions were used for Keithley (SMU-Model 2420) current–voltage (I–V) measurements. Recently, graphite and its derivatives such as graphite rods, plates, sheets, cloth, or paper are commonly used because graphite material is more valuable than simple carbon types. The graphite material is very rigid, brittle, thin and so far, non-toxic material (Yaqoob et al., 2021). The catalytic activity of a coin-sized urea fuel cell with graphite foil as the working and counter electrodes was first analyzed in 3 g of soil taken in a 3.14 cm^2^ area with urea fuel concentration of 0.5 g/mL for the cyclic voltammetry (CV) studies to check the studies are repeatable. Then, a single-chamber compost soil urea fuel cell (CS-UFC) was fabricated to see and compared the catalytic activity including the power density were compared which is 12 times higher than the coin cell (Magotra et al., 2021). An electrochemical study of CS-UFC was conducted using the coin-cell-type CR2032 system in previous studies (Magotra et al., 2020) as the reason behind that small scale is not possible to generate the higher power at large scale for commercial compost soil electrical applications. CV experiments were conducted due to high soil impedance. We employed small unit samples to form a single-chamber CS-UFC and performed soil studies to confirm whether the fuel cell performance and experimental studies are repeatable (Boggs et al., 2009; Kumar et al., 2018; Magotra et al., 2022).

However, for bacterial studies colony count study was performed with standard nutrient broth to verify the effect of the healthy growth of microbes on the samples with a urea concentration of 0.5 g/mL in the feed. First, urea was seeded into a 9 mL peptone saline diluent (PSD) for 2 h and incubated at a fixed ambient temperature. The inoculated PSD was diluted with fresh PSD 1:9, and the diluted soil sample suspension (100 μL) was directly distributed on the surface of the nutrient broth (N.B.) agar plates. After passing the 28 h, the bacteria growth was checked. The incubation temperature was 37°C.

### Electrochemical characterization

For the I–V measurements and electrical characterization, Kiteley’s high current source meter (SMU-Model-2420) interfaced with the RS-232 mode was used to study the different I–V parameters. The CV bipolar scans at a scan rate of 50 mV/s. Impedance Nyquist curve of EIS measurements consisting of the imaginary and real impedance components in a frequency range from 0 Hz to 10,000 Hz and for an applied alternating signal of 10 mV was measured. The electro-catalytic performance of compost for ammonium oxidation in a coin cell layout for electro-catalytic bio-battery formation was investigated using MPG-2 16-channel battery cycler (Bio-Logic Scientific Instruments, France). Here, the role of the bacteria in the carbon-rich compost soil CS-UFC sample was studied in comparison to an autoclaved sterilized sample of the CS-UFC treated at 121°C (to kill the bacteria). Then, I–V studies were performed to verify the role of the bacteria as electrocatalysts. Furthermore, temperature-dependent studies were performed at three different temperatures, 25, 40, and 55°C, using a Joe-Tech Oven (TC-ME-06, Seoul, Korea). In the I–V measurement studies, the cells need to be refueled to obtain a constant power output; thus, the cells require a continuous fuel supply, which is required for the regular performance of the CS-UFC. The refueling time is the ratio of the voltage across the load in the circuit to the maximum output voltage of the cell under the no-load conditions. Owing to the small size of the CS-UFC, previous studies increased the cell surface area from 3.14 to 15 cm^2^ to make it suitable for future commercial electrical applications as discussed above.

## Results and discussion

Figure 1 displays the schematic diagram and vision of this study for high power generation and the cleaning process initiated by the single chamber CS-UFC. Starting from the problem and reaches to the solution at the end. The vision of this paper will explain how the soil processes work in the CS-UFC. Eutrophication and toxicity affect contaminate soil and water on the earth, thus polluting the environment. This directly affects human health and endangers aquatic life due to the presence of excess chemicals and fertilizers. It has highly toxic chemicals, which lead to soil pollution making troubles in crop production. Presently, advanced microbial fuel cell devices perform multiple functions, such as removing toxicity, cleaning the environment, and green bioelectricity so if we find a solution to save the environment from these wastewaters it will be helpful to save the environment for future generations. While using urea-rich waste as fuel for power production for sustainable electricity generation.

**Figure 1:** The multifunctional role and vision of CS-UFC for the cleaning process and power generation.

Furthermore, Figure 2 displays Gr/Gr noble electrodes were used as current collector electrodes at the anode and cathode, which were separated by compost soil at the Center for single chamber CS-UFC. This fuel cell system is a completely membrane less system. This figure displays the schematic used for the I–V study for the commercial-sized design for continuous power generation from CS-UFC, wherein a computer setup and Keithley meter are connected to CS-UFC and used to regularly record data to verify the cycle and sustainability of the CS-UFC (US EPA, 2013).

**Figure 2:** Schematic of CS-UFC attached with Keithley for sustainable power generation.

For continuous device operation and for cleaning the excess nitrogen compounds from wastewater, a constant state is the most desirable, where the device behavior is irreversible, which helps to feed fuel to the device. Figure 2 reveals that when urea-rich fuel is supplied to a single chamber CS-UFC. The electron transfer begins. Compost soil itself works as a mediator, and separator in the CS-UFC to transfer the electrons directly from the cell toward the anode while the protons move toward the cathode. The arrows in the figure show the directions of movement of the electrons and protons shown in the working of CS-UFC (Logan, 2009; Jaiprakash, 2011; Javalkar and Alam, 2013; Jiang et al., 2016; Kumar et al., 2018).

The electrochemical characterization measurements (CV and EIS) were performed to study the Electrocatalytic activity of the CS-UFC. For fuel cells, the peak current and the onset potential are commonly used to evaluate the Electrocatalytic activity of a new catalyst toward any electro-oxidation or electro-reduction. It is well augmented in the case of fuel cells that the Electrocatalytic activity is studied by knowing about the peak current and the onset potential (Ding et al., 2016). The fuel cell works efficiently if the system is irreversible and it is the ideal condition for reducing the toxicity effects of the fuel by its total degradation. Efficient the degradation of fuel, the more will the cleaning of the environment as the toxicity of fuel reduces drastically with its degradation. EIS studies disclose the internal mechanism related to the electrochemical and kinetics behavior of the MFC. EIS measurements confirm the enhanced bio-electro-catalytic activity in MFC and the overall impedance decreases appreciably. These studies reveal the intrinsic electrochemical and kinetics mechanism of the CS-UFC. EIS measurements confirm the higher electro-catalytic activity in CS-UFC with urea as seen from CV measurements by showing that the overall impedance reduces significantly in comparison to the others.

Figures 3A–D displays the comparison of the catalytic activity of the samples. The optimization of the CS-UFC is addressed by considering peak current and onset potentials during the oxidation and reduction process. The Electrocatalytic activity was highest at a concentration of 0.5 g/mL of the urea fuel. This result indicated that urea fuel directly affects the compost soil for power generation. However, the redox potential peak for urea in the bipolar measurements fell in the range between 0 and ±0.6 V. It is similar to the values reported in the literature for urea, urine and near ammonium redox potentials (Bard et al., 2022). The general peaks shifted between 0 and ± 1 V, covering the range of water, urea, and urine to ammonium redox potential states. The value reported in the literature is consistent with the range of ±0.46 to ±0.49 V obtained for urea in the study (Ye et al., 2018). The overall reaction of urea occurred close to ±0.49 V, and this value is considerably lower than the 1.23 V required for the electrolysis; thus, theoretically, with the urea fuel cell. Figure 3A displays the comparison between D. I. water as a fuel in a liquid state vs. D.I. water with the addition of soil. The comparison shows the effect of the soil process in the solid state Figure 3B Urea fuel 0.5 g/mL in liquid state vs. CS-UFC with Urea fuel 0.5 g/mL displays the comparison between the urea fuel concentration of 0.5 g/mL fuel without and with the addition of soil for CS-UFC.

**Figure 3:** Bipolar CV studies show the performance of the liquid state and role of the carbon-rich compost soil **(A)** D. I. water (the liquid state) vs. D.I. water with the addition of soil, **(B)** Urea fuel 0.5 g/mL of in liquid state vs. CS-UFC with Urea fuel 0.5 g/mL **(C)** D. I. water with the addition of soil vs. CS-UFC with Urea fuel 0.5 g/mL **(D)** Comparison among 0.5 g/mL urea fuel in a liquid state, D. I. water with the addition of soil, CS-UFC with 0.5 g/mL urea fuel.

Figure 3A displays the comparison between D.I. water in the liquid state and D.I. water with the addition of soil. The figure clearly shows that the catalytic activity is enhanced in the addition of a soil sample. The comparison shows the effect of the soil process in the solid state.

Urea fuel 0.5 g/mL in liquid state vs. CS-UFC with Urea fuel 0.5 g/mL displays the comparison between the urea fuel concentration of 0.5 g/mL fuel without and with the addition of soil. Figure 3B displays the comparison between the liquid state with urea fuel and CS-UFC with urea fuel. The figure shows that owing to the redox potential difference, the soil state has a higher potential due to the direct effect of soil. Figure 3C displays that between D.I. water with the addition of soil sample and CS-UFC, the urea-fuel-based sample exhibited a higher redox potential. Figure 3D presents the comparison between soil with D.I. water with the addition of soil and CS-UFC. The results show the appreciable electro-catalytic activity of composts for CS-UFC in comparison to the CV of liquid urea solution which did not show any oxidation peak. Mild electro-oxidation peaks were observed in CS-UFC which can be due to the natural ammonium component present in composts. CV measurements with CS-UFC clearly show higher current density values in comparison with the other samples. For the continuous operation of a device for environment cleaning purposes, an irreversible state is the most desired state as it will help to feed the device continues with fuel filled with environmental toxins.

To verify the role of the compost soil (solid-state) in the ionic conductor of MFC, we have done further studies in comparison to the D. I. water (liquid state) as a pure electrolyte firstly. We took an ionic conductor (D. I. water + NaCl) mix with compost soil and analyzed with different NaCl concentrations used as fuel. We noticed that even the ionic conductor has a minute curve in the liquid state even using three different concentrations of NaCl (0.1, 0.2, and 0.3 g/mL). The liquid state has no role to raise the redox potential with NaCl. In the case of the addition of compost soil directly increases the catalytic activity as shown in the recorded CV curves. The redox potential is higher in support of the NaCl oxidation with the ionic conductor with the addition of (compost soil) in all concentrations of NaCl. The source of generating power in the compost soil is rich in organic matter, nutrient-rich and a thousand types of bacteria and enzymes present and working in themselves, which are responsible for the electrocatalyst activity and enhance the power after consuming the fuel. The compost soil is working as a source of ionic conductor, mediator, and source station for millions of bacteria. Here in our study, we are highlighting the role of the ionic conductor in power production and the solid state is a better option as compared to a liquid state.

From the above, all the compositions show the effective role of the soil and the redox potential is higher in all the samples with soil. The redox potential of CS-UFC is the highest rate and the soil process play here an important role. Both urea and ammonium ions are related to each other as sources of nitrogen and are used as fuel to accelerate the power generation process. The fuel cell device changed from a quasi-reversible to a constant state showing positive polarity. The study showing the electrochemical reaction on the active electrode surface, occurred due to a diffusion-controlled process, according to the Randel’s-Sevcik model. Thus, the system supports both the power generation purpose and the cleaning urea related waste materials. The potential redox peak for urea bipolar CV measurements was in the range of zero to ±1, which is similar to the values reported in the previous literature. The catalytic activities were in the ±0.1 to 0.6 V range for urea and ± 0.5 V range for the ammonium ions. Both urea and ammonium ions are related to each other as sources of nitrogen and are used as fuel to accelerate the power generation process (Bor-Yann et al., 2013; Sigurdarson et al., 2018; Wang et al., 2022).

Figures 4A–D displays the EIS difference among the samples followed by the CV studies from Figure 3. EIS is an efficient and non-destructive test for analyzing the bioelectrochemical processes of MFCs. The key factors limiting the output performance of an MFC can be identified by quantifying the contribution of its various internal parts to the total impedance. However, little attention has been paid to the measurement conditions and diagrammatic processes of the EIS for the fuel cell (Bisht and Chauhan, 2020). All of the peaks were recorded in the EIS measurements of compost samples, including the liquid state, and solid-state, either with or without soil. All impedance studies performed well with combinations as shown in the figure followed by CV data.

**Figure 4:** **(A)** Comparison of EIS liquid state and effect of carbon-rich compost soil. **(A)** D.I. water as a fuel in the liquid state vs. D.I. water with the addition of soil, **(B)** Urea fuel 0.5 g/mL in liquid state vs. CS-UFC with Urea fuel 0.5 g/mL **(C)** D.I. water with the addition of soil vs. CS-UFC with Urea fuel 0.5 g/mL **(D)** Comparison among 0.5 g/mL urea fuel in a liquid state, D.I water with the addition of soil, CS-UFC with 0.5 g/mL urea fuel, and circuit for EIS analysis (inset of **D**).

The comparative analyzes showed that the Electrocatalytic activity gradually increases, as the redox potential of CS-UFC with soil with 0.5 g/mL urea fuel is higher than that of soil without fuel in both voltage polarities. Higher redox potential curves have lower impedance values, and vice versa. The same trend was observed for all the samples depending upon the performance. Here EIS measurements were performed to investigate the electrochemical behavior of the compost soil. The high-frequency region has no semicircle in Figure 4 displays the charge transfer resistance (Rct) between the working electrode/electrolyte interfaces, which stems from the faradaic-redox reaction of the electrode. In the case of CS-UFC with urea, the value of Warburg impedance decreased remarkably, yielding increased diffusion-related kinetics during the ammonium oxidation reaction (Fricke et al., 2008).

We have tried to analyze EIS, and fitting of the observed EIS spectra using an equivalent circuit model was performed with ZsimpWin software. We have used the following circuit for EIS analysis (inserted in Figure 4D). The circuit consists of solution resistance (R_1_), charge transfer resistance (R_2_), a constant phase element (CPE_1_) and Warburg impedance (W_o_). The intersection between the real axis and the Nyquist plots at high frequency is attributed to Rs which is the intrinsic electrical resistance of the active electrode. A semicircle observed at high frequency to the mid-frequency region can be explained from the parallel combination of the Rct (charge transfer resistance) induced with redox reaction and CPE: constant phase element. From the EIS result, we also confirm the smaller charge transfer resistance of the additive added to the system compost soil, and graphite electrode than it is in liquid state or solid state, which matches well with the other experimental results present in the manuscript. For a soil MFC, the mass and electron transfer processes are relatively slow, and the system impedance value is high.

### Temperature dependence study

Figure 5A shows the temperature dependence using CV measurements for the CS-UFC with urea at 25, 40, and 55°C, respectively. Figures 5B,C shows the corresponding EIS measurement data which matches the CV trend fully. First starting from the room temperature at 25°C increases to 40°C, and then at last to 55°C to see the effect of temperature on the working of the CS-UFC device. The comparative studies show that electro-catalytic activity increases appreciably with the increase in temperature and is higher than 25°C. In the case of Electrocatalytic activity appreciably increased compared to that at room temperature at higher voltage polarities. The CV and EIS measurement trends are consistent with each other. The impedance trend at the highest redox potential corresponds to the lowest impedance or more vital Electrocatalytic activity at 55°C is highest than that at 40 and 25°C. The R_ct_ slowly decreases with increasing temperature, and the diffusion connected with the Warburg impedance is observed at room temperature, which disappears as the temperature increases. The impedance of CS-UFC with use decreased appreciably in comparison to the others leading to the conclusion that bio-electro-catalytic activity increases with the increase in temperature for the trend of CV observations (Behera et al., 2011). R_CT_ noticeably decreases significantly for CS-UFC. Warburg impedance which is related to the diffusion phenomenon also seems to decrease. Figure 5 clearly shows that the compost sample exhibits temperature-dependent behavior. Bio-electro-catalytic activity is found to increase with the increase in temperature which can be useful for applications at temperatures higher than room temperature.

**Figure 5:** Effect of temperature-dependent studies for standard sample CS-UFC at different temperatures. **(A)** Comparison among 25, 40, and 55°C. **(B)** EIS studies **(C)** Enlarged view of **(B)**.

### Cycle stability studies

The cyclic stability of the CS-UFC sample was performed with a single shot of 0.5 g/mL urea fuel tested over 600 cycles. In reality, such experiments are conducted at room temperature. The Device stability is also an essential factor that depends on the number of cycles, running stability, and how long the device may work. Figure 6A displays stability studies for 600 cycles showing that CS-UFC can be used as a long-term stable catalyst for fuel cells. Cyclic stability graphs are shown in Figure 6A. Figure 6B displays the results of the EIS studies before and after the 600-cycle test performed to check the effect of the impedance on the performance of CS-UFC. It proves the efficient repeatability of these results and the high stability of the CS-UFC just with the feeding of initial fuel. The results show that the cyclic stability of the device is sufficient for applications in both voltage polarities.

**Figure 6:** Cyclic stability of the compost soil with a single shot of fuel. **(A)** Cyclic stability plotted for 600 cycles. **(B)** EIS studies before stability and after stability for 600 cycles.

In this pursuit, energy storage devices such as fuel cells, which are mostly powered by organic compounds, can work as useful tools. Urea fuel cells available in the liquid state are not sustainable and portable. However, soil-based MFC uses natural bacteria or secreted enzymes to break down the fuel, typically to generate electricity from the soil. In MFCs, bacteria and enzymes act as biocatalysts to produce electricity. Until now, the reported liquid-state MFCs associated with safety concerns mainly related to toxicity, shifting, leakage, handling and degrading fastely in the liquid state (Kumar et al., 2018). Moreover, additional precautions are needed to prevent exposure to gaseous NH_3_ due to the volatilization of the liquid fuel. Therefore, solid-state materials like soil compost are preferred to overcome the risk, as mentioned above for stable behavior.

Among elements of urine, urea is most of all. Urine, wastewater and nitrogen fertilizer are suitable fuels for MFCs in the future. We need to study the role of urea as the main element of urine, wastewater and nitrogen fertilizer. Moreover, it is advantageous for the soil-based system to go through the natural cleaning processes by following nitrification and denitrification in the nitrogen cycle by ammonification to nitrogen (N_2_) formation in soil. The soil itself is a source of many bacteria and microorganisms in aerobic and anaerobic forms. Urea and ammonium are elements of nitrogen fertilizer also. If urea and ammonium as fuel in the land will obtain electrical power and remove fertilizer (Wang et al., 2017; Kumar et al., 2018; Magotra et al., 2020; Senthilkumar and Naveen Kumar, 2020; Kim et al., 2022; Magotra et al., 2022).

Urea when comes in contact with the soil while hydrolysis releases urease enzymes working as a catalyst with bacteria. Therefore, soil systems can be a neutral medium to transport electrons and protons easily in an eco-friendly medium for power generation. Power generation from urea as fuel is shallow in the liquid state, as shown in various studies done previously. The conventional charge separator, like a membrane, Nafion routinely used in the liquid type multiple chambers MFC, is expensive. Therefore, the soil advantage here soils themselves work as a charge separator. It is a purely microbial system the soil itself works as a separator, mediator, and ionic conductor to promote electrons and protons in the soil-based single-chamber MFC (Bor-Yann et al., 2013; Wang et al., 2017; Kumar et al., 2018; Magotra et al., 2022).

Figure 7A shows the strength of the fuel cell with urea fuel concentration ranging from 0.1 to 0.5 g/mL. The highest catalytic activity was observed at 14 h with the inert Gr/Gr electrodes. Then, the device stability was checked after adding 0.5 g/mL urea fuel at regular intervals of time. The generated power density was 55.26 mW/m^2^, as shown in Figure 7B. Figure 7C displays the effects of urea concentration on the power density of the fuel cell (Lan, 2010). The Electrocatalytic activity and electro-oxidation of urea exhibit the same trend for both the polarities of the redox potential. For the urea fuel concentration of 0.5 g/mL, a maximum oxidation peak generates the highest power as shown in Figure 7C. Thus, the power density is concentration-dependent, and the highest Electrocatalytic activity showed for the highest urea fuel concentration. Thus, from this single chamber CS-UFC studies show the role of soil processes and their direct effects on power generation (Xu et al., 2016). The role of the addition of urea as a fuel is to provide nitrogen with nitrification and denitrification in our manuscript. When using urea as fuel for single-chamber CS-UFC (Bor-Yann et al., 2013; Wang et al., 2017). Compost soil itself is loaded with ions and exhibits electronic behavior due to aerobic and anaerobic bacteria and enzymes. One gram of soil contains more than 1,000–2,000 types of bacteria. Moreover, both urea, and ammonium are the main sources of nitrogen. Urea is working as food for the bacteria in the soil and compost soil has its role in the CS-UFC (Simeon et al., 2020).

**Figure 7:** Gr/Gr Electrodes, Keithley I–V measurement data using 0.5 g/mL carbon-rich compost. **(A)** Urea fuel concentration ranges from 0.1 to 0.5 g/mL with single-chamber CS-UFC. **(B)** The polarization curve of CS-UFC. **(C)** Concentration ranges from 0.1 to 0.5 g/mL. **(D)** Effect of PH stability without and with soil using 0.5 g/mL of standard fuel.

The role of the addition of urea is to provide nitrogen with nitrification and denitrification in our manuscript. When using urea as fuel for single-chamber CS-UFC (Wang et al., 2017). Compost soil itself is loaded with ions and exhibits electronic behavior due to aerobic and anaerobic bacteria and enzymes. One gram of soil contains more than 1,000–2,000 types of bacteria. Moreover, both urea, and ammonium are the main sources of nitrogen. Urea is working on its role in the CS-UFC (Zhang et al., 2021).

The pH sustainability studies also performed for CS-UFC were confirmed while supplying standard urea fuel 0.5 g/mL at the beginning of the first running cycle (0–28 h). The pH of the compost was 9.2 and slowly increased to 9.7 in the fuel cell while refueling continually every 28 h as shown in Figure 7D. We recorded the pH data with a pH meter (Apera PH700 benchtop lab pH meter) used to perform the studies and continuously diagnose the study for max from (0 to 140) hrs. The role of pH in the liquid and solid states of the compost fuel cell is crucial for power output. The pH studies of liquid state urea fuel 0.5 g/mL without the addition of compost soil in comparison with the CSUFC standard sample showed that pH shows an effect from the liquid to solid state. These are due to the addition of soil, which helps enhance power production (Lee et al., 2004). Due to the addition of nitrogen in the soil, the chemical reaction enhances the pH from 6.5 to an alkaline pH in the range of 8–9. The *V*_max_ for the high-affinity response reaction (N_2_O → NO → N_2_) showed a relatively small peak at pH 6.5, followed by first a decline and then a sharp increase in the pH to 9.5 to 9.7. Urea is food for the bacteria; urea stimulates bacteria to release urease. When urea was hydrolysed, it generates ammonia, and ammonium ions (NH_4_^+^ ions). Compost soil performs ammonification through nitrification and denitrification processes to reach release (N_2_) as the last product while supplying protons and electrons (Žalnėravičius et al., 2022).

The proposed single-chamber CS-UFC employs industrial wastewater, urea, and urine-rich wastewater as the catalyst for soil bacteria and enzymes, which is economical, for power generation.

Nevertheless, compared to the 0.5 g/mL urea fuel fed to the CS-UFC, the power generation is enhanced which shows the effect on the pH study. The increase in the pH is due to proton consumption and OH (hydroxyl group) generation by the anodic and cathodic side reactions in the soil, which mostly indicates the effect of different types of bacteria and enzymes (He et al., 2008).

Figures 8A,B displays the sustainability study for the power density, with the maximum peak at 14 h and the single cycle was completed at (0–28) hour cycle (Cabrera et al., 1991). The I–V measurement studies represent the fuel cell sustainability, while the power generation and pH exhibit stable behavior as we optimized for 224 h while supplying the fuel continually. The results of the sustainability studies was shown in Figure 8A. The commercial fuel cell was refueled several times after every 28 h. accordingly. The power generation was monitored to assess the fuel cell’s sustainability in comparison study to pH stability in with working of CS-UFC performance. The results show that the normal stable functioning of the single chamber CS-UFC continues until we supplied fuel to the device (Tang et al., 2014).

**Figure 8:** Gr/Gr Electrodes, Keithley I–V measurement data for sustainability studies using carbon-rich compost with 0.5 g/mL fuel. **(A)** Sustainability study for CS-UFC for 224 h. **(B)** pH sustainability during the working of CS-UFC.

To study the urea consumption, urea fuel 0.5 g/mL in the liquid state was injected at regular intervals of time and its current and power densities were calculated using Keithley (I-V) meter. We injected the urea fuel and left it for activation. The sample was activated and optimized which showed maximum peak power at 14 h in a single cycle, and then, the fuel degraded and power decreased. After refueling, the same trend was observed in the 2nd cycle. This indicates that CS-UFC devices consume urea fuel and generate power.

In the analysis of the CS-UFC device pH study, sustainability was measured at room temperature until 224 h in comparison to the working of a fuel cell, and the sustainability of CS-UFC was investigated. The results show that pH in the liquid state decreased, while in the power generation process in compost, the soil starts higher up taking fuel. A balanced system was established within the range of pH 9.2–9.7 in the compost-based system. A high pH value does not affect electricity generation due to the buffer effects of the bacterial activities in the fuel cell. Figure 8B shows the pH difference between the liquid and solid states; the solid state has a stable and higher pH than the liquid state, which is helpful for electricity generation for compost fuel cells that are regularly optimized and monitored (Cabrera et al., 1991).

To verify the effect of enzymes and bacteria for power generation on single chamber CS-UFC. Here we performed experiments with standard NB to demonstrate the effect of microbe cultivation on the power generation performance of compost samples at regular intervals of time as shown in Figures 9A–D. At the beginning of Figure 9A, the bacterial study was performed using two samples for comparison: one was prepared with a standard compost sample containing 0.5 g/mL urea fuel composed of a live bacteria sample (Yin et al., 2011). The other was an identical standard sample, albeit it was autoclaved at a temperature of 121 C^0^ to kill all of the bacteria and enzymes using autoclaved sterilization workstation (Bernhard, 2010). The comparison results confirmed the role of the bacteria and enzymes present in the live bacteria sample. The cultivation of the microbes is start between 28 h, and it starts to increase gradually with bacterial growth visible on the plates shown in Figure 9A. However, the results confirm the no negligible role of the microorganisms after 28 h. In the case of the autoclaved sample, there is no bacterial growth or enzyme activity throughout the experiment shown in Figure 9B. Thus, this study indicated the role of urea fuel in power generation due to the influential role of single-chamber CS-UFC. The similarity in the results obtained from bacterial studies and I-V measurements suggests that bacteria and enzymes played an essential role in power generation (Liu et al., 2014). This confirms the role of compost as a biocatalyst. As shown in Figure 9C, the same bacterial study effect was repeated other with Keithley (I-V) measurements using 0.5 g/mL fuel for CS-UFC. The results verified that the effects of the live urease enzymes and bacteria increased the sustained power density to 55.26 mW/m^2^. In comparison, the power density of the autoclaved sample was minute to 1.2 mW/m^2^ owing to the absence of any bacteria. Thus, the CV and I-V studies results are consistent and confirm the roles of the enzymes and bacteria for the power generation in the single chamber CS-UFC (Kumar et al., 2018; Shaw et al., 2020). In this paper, we demonstrated the single chamber CS-UFC can be a neutral medium to transport electrons and protons easily in an eco-friendly medium due to refueling fuel for high power generation. Presently, advanced CS-UFC performs multiple functions, such as removing toxicity, cleaning the environment, and green bioelectricity.

**Figure 9:** Effect of the bacterial study for compost soil coin samples: **(A)** growth of the bacterial colonies present and **(B)** growth of colonies absent. **(C)** The I–V data between the standard compost sample and autoclaved sample on power generation. **(D)** Real photos of CS-UFC with and without microbe growth.

From Figure 9D real plates were photographed, and the soil bacteria and autoclaved samples were examined for a longer time up to 224 h. The results show that CS-UFC affords enhanced energy and sustainability due to the advantageous effects of different types of soil bacteria and enzymes (anaerobic and aerobic). An alkaline medium was used to perform the urea electrolysis for carbon-neutral bioelectricity generation (Barakat et al., 2018).

Our study results show that the combined mechanism of compost soil and urea fuel cell enhances power generation as urea fuel is dissolved in a liquid state to facilitate its uptake and catalysis by soil bacteria and enzymes (Urbańczyk et al., 2016).

Soil is a well-known electro-catalyst. Similar to bacteria and enzymes, the soil may catalyze the oxidation of urea. Due to the addition of the urea nitrogen source in the soil, the chemical reaction enhances the ph. Furthermore, the V_max_ for the high-affinity response of the (N_2_O → NO→N_2_) reaction exhibited a relatively small peak, followed by a decline and then a sharp increase. Urea is always a portion of food for the bacteria, and it stimulates bacteria to release urease (Ghaly and Ramakrishnan, 2013). When urea is hydrolyzed, it generates ammonia and transforms to ammonium ions (NH_3_ to NH_4_ ions), which do not volatilize.

Compost soil in operation performs ammonification *via* the nitrification and denitrification processes to release the last product (N_2_) while supplying electrons and protons. When urea is hydrolyzed, the urease enzyme is released in the soil at a faster rate than that in liquid; subsequently, ammonia and ammonium ions (NH_4_ + ions) are generated. Moreover, ammonification and volatilization lead to nitrification and denitrification processes (Li et al., 2018).

Reaction 1 (NH_3_ + O_2_ + 2e^−^ → NH_2_OH + H_2_O): Conversion of urea to ammonia and then hydroxylamine, which is catalyzed by enzymes to ammonia monooxygenase. Reaction 2 (NH_2_OH + H_2_O → NO_2_^−^ + 5H^+^ + 4e^−^): Hydroxylamine is converted to nitrite, which is catalyzed by enzymes to hydroxylamine oxidoreductase (Jiang et al., 2016).

Bacteria oxidize urea to nitrogen gas and carbon dioxide, generating ammonia or transforming to ammonium ions, which are converted to carbonic acid C.O. (OH)_2_ or carbamate, as reported in the literature. Ammonification transforms *Nitrosomonas and Nitrobacter* to NO_3_ (nitrate) or directly NO_2_ (nitrite) *via* nitrification, eventually producing nitrogen (N_2_) (Ye et al., 2018).

Therefore, compost soil systems are a natural medium for easily transporting electrons and protons in an eco-friendly and non-toxic manner for power generation. This study confirmed the profound effect of urea on power generation using the CS-UFC. The focus is to generate power from the CS-UFC in the coming future using waste like urea-rich wastewater, urine, and industrial wastewater, which contain considerable amounts of urea (Rysgaard et al., 1996).

## Conclusion

This study demonstrated the multifunctional role of CS-UFC. CS-UFC can generate power using urea as fuel. Moreover, it can produce electricity, reduce eutrophication, and toxicity effect, which contaminates soil and groundwater by consuming urea-rich wastewater from water and soil pollution and contribute to environmental cleanup. The urea fuel concentration of 0.5 g/mL in soil was found to be optimal, yielding a power density of 55.26 mW/m^2^. Furthermore, this device was shown to be sustainable for electricity generation. It exploits different types of energy-generating soil bacteria and enzymes already present in the soil. Additionally, it can combat water and soil pollution. This study optimized the advancements of single CS-UFC by providing a sustainable, eco-friendly, and economical energy generation technology with plenty of scope for future research. On the other hand, for enhancing the power at a large scale, our group working on the multiple stacks in series and parallel for enhancing the powerhouse in bulk systems in the coming future for finding a solution for green energy applications for running the electricity-based devices at small and large scale.

## Data availability statement

The raw data supporting the conclusions of this article will be made available by the authors, without undue reservation.

## Author contributions

VM and HJ conducted the main work of this article, including plotting the figures, and drafting the manuscript. TK and SL provided the suggestions. All authors approved the final manuscript.

## Funding

This research project sponsored by the Basic Science, Research Program through the National Research Foundation of Korea (NRF), funded by the Ministry of Education, Science and Technology (2016R1A6A1A03012877, 2022R1F1A1066650).

## Conflict of interest

The authors declare that the research was conducted in the absence of any commercial or financial relationships that could be construed as a potential conflict of interest.

## Publisher’s note

All claims expressed in this article are solely those of the authors and do not necessarily represent those of their affiliated organizations, or those of the publisher, the editors and the reviewers. Any product that may be evaluated in this article, or claim that may be made by its manufacturer, is not guaranteed or endorsed by the publisher.

## References

[ref1] AdegokeT. O. (2022). Tae-il Moon, and Hyun-Hwoi Ku, ammonia emission from sandy loam soil amended with manure compost and urea, applied. Biol. Chem. 65, 1–9.

[ref2] AngarY.EddineN. (2015). Influence of the anode nature in the ammonium electro-oxidation. Rev. Roum. de Chime 60, 1039–1046.

[ref3] AngladaA.IbanezR.UriegasA.InmaculadaO. (2010). Electrochemical oxidation of saline industrial wastewaters using boron-doped diamond anodes. Catal. Today 151, 178–184. doi: 10.1016/j.cattod.2010.01.033

[ref4] BarakatN. A. M.AlajamiM.GhouriZ. K.Al-MeerS. (2018). Co-Ni/nanoparticles/CNT composite as effective anode for direct urea fuel cells. Int. J. Electrochem. Sci. 13, 4693–4699.10.3390/nano8050338PMC597735229772710

[ref5] BardA. J.FaulknerL. R.WhiteH. S. (2022). Electrochemical Methods: Fundamentals and Applications. John Wiley & Sons Ltd.

[ref6] BaveyeP. C.SchneeL. S.BoivinP.LabaM.RadulovichR. (2020). Soil organic matter research and climate change: merely re-storing carbon versus restoring soil functions. Front. Environ. Sci. 8:579904

[ref7] BeheraM.MurthyS. S. R.GhangrekarM. M. (2011). Effect of operating temperature on the performance of microbial fuel cell. Water Sci. Technol. 64, 917–922. doi: 10.2166/wst.2011.70422097080

[ref8] BernhardA. E. (2010). The nitrogen cycle: processes, players, and human impact. Nat. Educ. Knowl. 2:12.

[ref9] BishtN.ChauhanP. S. (2020). Excessive and disproportionate use of chemicals cause soil contamination and nutritional stress. Soil Contamin. Threats Sustain. Solutions, 1–10. doi: 10.5772/intechopen.94593

[ref10] BoggsB. K.KingR. L.BotteG. G. (2009). Urea electrolysis: direct hydrogen production from urine. Chem. Commun. 32, 4859–4861. doi: 10.1039/b905974a, PMID: 19652805

[ref11] Bor-YannC.Shi-QiL.Jhao-YinH.Tz-JauS.Yu-MinW. (2013). Reduction of carbon dioxide emission by using microbial fuel cells during wastewater treatment. Aerosol Air Qual. Res. 13, 266–274. doi: 10.4209/aaqr.2012.05.0122

[ref12] BurkeL. D.NugentP. F. (1983). The electrochemistry of gold II: the electrocatalytic behaviour of the metal in aqueous media. Gold Bull. 31, 39–50.

[ref13] CabreraM. L.KisselD. E.BockB. R. (1991). Urea hydrolysis in soil: effects on urea concentration and soil pH. Soil Biol. Biochem. 23, 1121–1124. doi: 10.1016/0038-0717(91)90023-D

[ref14] CalikogluU.KoksalM. A. (2022). Green electricity and renewable energy guarantees of origin demand analysis for Türkiye. Energy Policy 170:113229. doi: 10.1016/j.enpol.2022.113229

[ref15] ChoK.HoffmannM. R. (2017). Molecular hydrogen production from wastewater electrolysis cell with multi-junction BiO_x_/TiO_2_ anode and stainless steel cathode: current and energy efficiency. Appl. Catal. B Environ. 202, 671–682. doi: 10.1016/j.apcatb.2016.09.067

[ref16] DingK.ChenY.ZhaoJ.ZhangY.WeiB. (2016). The influence of potential sweep cycle number on the electrocatalytic activity of the boiled PdO/graphene for ethanol oxidation reaction (EOR). Int. J. Electrochem. Sci. 11, 9481–9490. doi: 10.20964/2016.11.47

[ref17] FrickeK.HarnischF.SchroderU. (2008). On the use of cyclic voltammetry for the study of anodic electron transfer in microbial fuel cells. Energy Environ. Sci. 1, 144–147. doi: 10.1039/b802363h

[ref18] GhalyA. E.RamakrishnanV. V. (2013). Nitrification of urea and assimilation of nitrate in saturated soils under aerobic conditions. Am. J. Agric. Biol. Sci. 8, 330–342. doi: 10.3844/ajabssp.2013.330.342

[ref19] HeZ.HuangY.ManoharA. K.MansfeldF. (2008). Effect of the electrolyte P.H. on the rate of the anodic and cathodic reactions in an air cathode microbial fuel cells. J. Biochem. 74, 78–82.10.1016/j.bioelechem.2008.07.00718774345

[ref20] HuazhangZ.ZhangY.ZhaoB.ChangY.LiZ. (2012). Electrochemical reduction of carbon dioxide in an MFC–MEC system with a layer-by-layer self-assembly carbon nanotube/cobalt phthalocyanine modified electrode. Environ. Sci. Technol. 46, 5198–5204. doi: 10.1021/es300186f, PMID: 22475021

[ref21] JaiprakashV. (2011). *Novel cowdung based microbial fuel cell*. United States Patent Application Publication, U.S 20110135966A1.

[ref22] JavalkarP. D.AlamJ. (2013). Comparative study on sustainable bioelectricity generation from a microbial fuel cell using bio-waste as fuel. Int. J. Sci. Res. Publ. 3, 1–6.

[ref23] JiangY.-B.ZhongW. H.HanC.DengH. (2016). Characterization of electricity generated by soil in microbial fuel cells and the isolation of soil source exoelectrogenic bacteria. Front. Microbiol. 7:1776. PMID: 2787716810.3389/fmicb.2016.01776PMC5099896

[ref24] KapałkaA.FierroS.FrontistisZ.KatsaounisA.NeodoaS.FreyO.. (2011). Electrochemical oxidation of ammonia (NH_4_+/NH_3_) on thermally and electrochemically prepared IrO2 electrodes. Electr. Acta 56, 1361–1365. doi: 10.1016/j.electacta.2010.10.071

[ref25] KimO.-H.ChoiH. J.KangS. Y.JangG. Y.KaruppannanM.ParkJ. E.. (2022). Towards outstanding performance of direct urea fuel cells through optimization of the anode catalyst layer and operating conditions. J. Electroanal. Chem. 921:116661. doi: 10.1016/j.jelechem.2022.116661

[ref26] KumarS.MagotraV. K.JeonH. C.KangT. W.InamdarA. I.AqueelA. T.. (2018). Multifunctional ammonium fuel cell by using compost as an oval electrocatalyst. J. Power Sources 402, 221–228. doi: 10.1016/j.jpowsour.2018.09.041

[ref27] LanR. (2010). Shanwen Tao, and John TS Irvine, a direct urea fuel cell–power from fertiliser and waste. Energy Environ. Sci. 3, 438–441. doi: 10.1039/b924786f

[ref28] LeeH. K.ChoiH. Y.ChoiK. H.ParkJ. H.LeeT. H. (2004). Hydrogen separation using electrochemical method. J. Power Sources 132, 92–98. doi: 10.1016/j.jpowsour.2003.12.056

[ref29] LiY.ChapmanS. J.NicolG. W.YaoH. (2018). Nitrification and nitrifies in acidic soils. Soil Biol. Biochem. 116, 290–301. doi: 10.1016/j.soilbio.2017.10.023

[ref31] LiuC. W.SangY.ChenB. C.LaiH.-Y. (2014). Effects of nitrogen fertilizers on the growth and nitrate content of lettuce. Int. J. Public Health 11, 4427–4440.10.3390/ijerph110404427PMC402500024758896

[ref32] LoganB. E. (2009). Exoelectrogenic bacteria that power microbial fuel cells. Nat. Rev. Microbiol. 7, 375–381. doi: 10.1038/nrmicro211319330018

[ref33] MagotraV. K.KangT. W.Aqueel AhmedA. T.InamdarA. I.ImH.GhodakeG.. (2021). Effect of gold nanoparticles laced anode on the bio-electro-catalytic activity and power generation ability of compost-based microbial fuel cell as a coin cell-sized device. Biomass Bioenergy 152:106200. doi: 10.1016/j.biombioe.2021.106200

[ref34] MagotraV. K.KangT. W.KimD. Y.InamdarA. I.WalkeP. D.LeeS. J.. (2022). Urea fuel cell using cow dung compost soil as a novel biocatalyst for power generation applications. Energy 239:122357. doi: 10.1016/j.energy.2021.122357

[ref35] MagotraV. K.LeeS. J.InamdarA. I.KangT. W.WalkeP. D.HoganS. C.. (2021). Development of white brick fuel cell using rice husk ash agricultural waste for sustainable power generation: a novel approach. Renew. Energy 179, 1875–1883. doi: 10.1016/j.renene.2021.08.003

[ref36] MagotraV. K.LeeS. J.KangT. W.InamdarA. I.KimD. Y.ImH.. (2022). High power generation with reducing agents using compost soil as a novel electrocatalyst for ammonium fuel cells. Nano 12:1281. doi: 10.3390/nano12081281, PMID: 35457989PMC9029104

[ref37] MagotraV. K.SunilK.KangT. W.InamdarA. I.AqueelA. T.ImH.. (2020). Compost soil microbial fuel cell to generate power using urea as fuel. Sci. Rep. 10:4154. doi: 10.1038/s41598-020-61038-7, PMID: 32139783PMC7058052

[ref39] PerezG.SaizJ.IbanezR.UrtiagaA. M. (2012). Ortiz, assessment of the formation of inorganic oxidation by-products during the electrocatalytic treatment of ammonium from landfill leachates. Water Res. 46, 2579–2590. doi: 10.1016/j.watres.2012.02.015, PMID: 22386329

[ref40] Piche-ChoquetteS.ConstantP. (2019). Molecular hydrogen a neglected key driver of the soil biological processes. Appl. Environ. Microbiol. 85, 1–19. doi: 10.1128/AEM.02418-18PMC641437430658976

[ref41] RollinsonA. N.RickettG. L.LangtonA. L.DupontV.TwiggM. V. (2011). Hydrogen from urea water and ammonia water solutions. Appl. Catal. B Environ. 106, 304–315. doi: 10.1016/j.apcatb.2011.05.031

[ref42] RysgaardS.Risgaard-PetersenN.SlothN. P. (1996). “Nitrification, denitrification, and nitrate ammonification in sediments of two coastal lagoons in Southern France” in Coastal Lagoon Eutrophication and ANaerobic Processes (C.L.E.AN.). Developments in Hydrobiology. eds. CaumetteP.CastelJ.HerbertR. (Dordrecht: Springer), 133–141.

[ref43] SenthilkumarK.Naveen KumarM. (2020). “Generation of bioenergy from industrial waste using microbial fuel cell technology for the sustainable future” in Refining Biomass Residues for Sustainable Energy and Bioproducts: Technology, Advances, Life Cycle Assessment, and Economics. eds. Praveen KumarR.JegannathanK. R.EdgardG.BaskarG. (Cambridge, MA: Academic Press), 183–193.

[ref44] ShawD. R.AliM.KaturiK. P.GralnickJ. A.ReimannJ.MesmanR.. (2020). Extracellular electron transfer-dependent anaerobic oxidation of ammonium by anammox bacteria. Nat. Commun. 11, 1–12.3234597310.1038/s41467-020-16016-yPMC7188810

[ref45] SigurdarsonJ. J.SvaneS.KarringH. (2018). The molecular processes of urea hydrolysis to ammonia emissions from agriculture. Rev. Environ. Sci. Biotechnol. 17, 241–258. doi: 10.1007/s11157-018-9466-1

[ref46] SimeonM. I.AsoiroF. U.AliyuM.RajiO. A.FreitagR. (2020). Polarization and power density trends of a soil-based microbial fuel cell treated with human urine. Int. J. Energy Res. 44, 5968–5976. doi: 10.1002/er.5391

[ref47] SinghJ.KunhikrishnanA.SaggarS.BolanN. S. (2013). Impact of urease inhibitor on ammonia and nitrous oxide emissions from, cores receiving urea, temperature pasture soil fertilizer and cattle urine. Sci. Total Environ. 465, 56–63. doi: 10.1016/j.scitotenv.2013.02.018, PMID: 23473618

[ref30] TangJ.LiuT.YuanY.ZhuangL. (2014). Effective control of bioelectricity generation from a microbial fuel cell by logical combinations of pH and temperature. Sci. World J. 2014, 1–7. doi: 10.1155/2014/186016PMC397285224741343

[ref48] TengY.YongfengX. U.WangX. (2019). Peter Christie function of biohydrogen metabolism and related microbial communities in environmental bioremediation. Front. Microbiol. 10:106. doi: 10.3389/fmicb.2019.00106, PMID: 30837956PMC6383490

[ref49] ThulasinathanB.JayabalanT.ArumugamN.Rasu KulanthaisamyM.KimW.KumarP.. (2022). Wastewater substrates in microbial fuel cell systems for carbon-neutral bioelectricity generation: an overview. Fuel 317:123369. doi: 10.1016/j.fuel.2022.123369

[ref50] UrbańczykE.SowaM.SimkaW. (2016). Urea removal from aqueous solutions-a review. J. Appl. Electrochem. 46, 1011–1029. doi: 10.1007/s10800-016-0993-6

[ref380] US EPA (2013). Composting at home. Available at: https://www.epa.gov/recycle/composting-home (Accessed February 14, 2023).

[ref51] VaishaliS.DasD. (2019). “Potential of hydrogen production from biomass” in Science and Engineering of Hydrogen-Based Energy Technologies. Amsterdam: Elsevier Inc., 123–164.

[ref52] VraghavuluS.MohanS. V.GoudR. K.SarmaP. N. (2009). Effect of anodic pH microenvironment on microbial fuel cell(MFC) performance in concurrence with aerated and ferricyanide catholyte. Electrochem. Commun. 11, 371–375. doi: 10.1016/j.elecom.2008.11.038

[ref53] WangC.-T.LiaoF.-Y.LiuK.-S. (2013). Electrical analysis of compost solid phase microbial fuel cell. Int. J. Hydrog. Energy 38, 11124–11130. doi: 10.1016/j.ijhydene.2013.02.120

[ref54] WangH.LongX.SunY.WangD.WangZ.MengH.. (2022). Electrochemical impedance spectroscopy applied to microbial fuel cells: a review. Front. Microbiol. 13:973501. doi: 10.3389/fmicb.2022.97350135935199PMC9355145

[ref55] WangL.XieB.GaoN.MinB.LiuH. (2017). Urea removal coupled with enhanced electricity generation in single-chambered microbial fuel cells. Environ. Sci. Pollut. Res. 24, 20401–20408. doi: 10.1007/s11356-017-9689-7, PMID: 28707242

[ref56] XuW.ZuchengW.TaoS. (2016). Urea-based fuel cells and electrocatalysts for urea oxidation. Energ. Technol. 4, 1329–1337. doi: 10.1002/ente.201600185

[ref57] YaqoobA. A.IbrahimM. N. M.UmarK. (2021). “Electrode material as anode for improving the electrochemical performance of microbial fuel cells” in Energy Storage Battery Systems-Fundamentals and Applications. eds S. Haider, A. Haider, M. Khodaei and L. Chen (IntechOpen Ltd.).

[ref58] YeK.WangG.CaoD.WangG. (2018). Recent advances in the electro-oxidation of urea for direct urea fuel cell and urea electrolysis. Top Curr. Chem. 376:42. doi: 10.1007/s41061-018-0219-y, PMID: 30367274

[ref59] YinD.ZhouS.-G.ChenQ.ZhaoB.YuanY.ZhuangL. (2011). Enhanced anaerobic degradation of pollutants in a soil microbial fuel cell. Chem. Eng. J. 172, 647–653.

[ref60] ŽalnėravičiusR.PaškevičiusA.Samukaitė-BubnienėU.RamanavičiusS.VilkienėM.MockevičienėI.. (2022). Microbial fuel cell based on nitrogen-fixing Rhizobium anhuiense bacteria. Biosensors 12:113. doi: 10.3390/bios12020113, PMID: 35200373PMC8869864

[ref61] ZhangX.LiX.ChenX.SunY.ZhaoL.HanT.. (2021). A nitrogen supplement to regulate the degradation of petroleum hydrocarbons in soil microbial electrochemical remediation. Chem. Eng. J. 426:131202. doi: 10.1016/j.cej.2021.131202

[ref62] ZiyauddinU.PathrikarA. K. (2013). The future of energy bio battery. Int. J. Eng. Res. Technol. 2, 99–111.

